# Cigarette Smoke Regulates the Expression of EYA4 via Alternation of DNA Methylation Status

This article has been retracted.

**DOI:** 10.1155/2022/5032172

**Published:** 2022-05-14

**Authors:** Bader O. Almutairi, Mikhlid H. Almutairi, Abdulwahed F. Alrefaei, Daoud Ali, Saad Alkahtani, Saud Alarifi

**Affiliations:** Department of Zoology, College of Science, King Saud University, P.O. Box: 2455, 11451 Riyadh, Saudi Arabia

## Abstract

Cigarette SMOKE (CS) considerably contributes to causing some diseases such as cancer, and it has a role in the alternation of gene expression through several mechanisms including epigenetics modification, particularly DNA methylation. *EYA4* is one of the genes, that whose expression has been dysregulated in lung, colon, bladder, and breast cancer, leading to tumor progression. The alternation of DNA methylation levels has been implicated in regulating the expression of the *EYA4* gene. Thus, in this study, we have shown the effect of CS on the DNA methylation level of the *EYA4* promoter region as well as the methylation level on *EYA4* expression. To determine the level of DNA methylation on the promoter region of the *EYA4* gene, we have employed the bisulfite conversion treatment followed by the Sanger Sequence for 100 DNA samples taken from Saudi people (50 smokers and 50 nonsmokers). We found that 26% of DNA extracted from smoker samples is methylated, while there was no methylation identified in nonsmoker samples. Also, using the demethylating agents such as AZA on LoVo and Caco-2 cancer cell lines causes induction of transcription level of *EYA4*, implying the possible mechanism of DNA methylation in the upregulation of *EYA4*. These findings suggest the possible mechanism of CS in controlling the expression of *EYA4* via changing the status of DNA methylation.

## 1. Introduction

Cigarette smoke (CS) is the most prevalent cause of death and disease in the world [1]. CS may negatively affect nearly all organs of the body, accelerate the process of organ aging, and consequently lead to various disease, such as cardiovascular diseases [1], chronic obstructive pulmonary disease [2], and cancers [3]. Clinical studies have illustrated that CS can trigger several aging-related changes, from cell phenotype to gene expression and epigenetic regulation, in the respiratory system [4], as well as the ability to induce oxidative damage, inflammation, immune changes, genetic alterations [5], and single-nucleotide polymorphism (SNP) alternations [6]. Thus, understanding the mechanism of smoking and its contribution of causing chronic illness is a crucial for the discovery of therapeutic targets [7]. Few studies have been conducted on epigenetic mechanisms including DNA methylation, showing a possible role of CS in regulation of DNA methylation [8] that could lead to remarkable changes in gene transcription, resulting in diseases development [9–11].

Epigenetics, including DNA methylation, has been implicated in causing several diseases such as neuroblastoma [12], breast cancer [13], colon cancer [14], and liver cancer [14], via silencing tumor suppressor genes [15] and inducing oncogenes [12]. Recent studies have shown that the alternation of DNA methylation is a leading cause of colon cancer and being considered as biomarkers [16]. It is noteworthy that several environmental factors can negatively affect the epigenetic mechanisms including DNA methylation [8], especially CS, air pollution, and dietary changes [8].

One of the specific genes which has been regulated by alternation of DNA methylation is *EYA4* [17, 18], and it belongs to eyes absent gene family (EYA), playing a major role in the mediation of DNA repair, cell apoptosis, angiogenesis, and tumor growth [19, 20]. EYA protein harbors different domains, including transcriptional activation, protein tyrosine phosphate, and threonine phosphate, and its conserved C-terminal domain carrying 270 amino acids, while less likely conserved N-terminal having a vary amino acids between 266 and 320 [21]. Translational level of EYA, particularly protein-protein interaction domain involves in the binding site of SIX and DACH protein [22]. Interestingly, disruption of *EYA4* expression was implied to contribute to cancer progression including lung cancer [23], hepatocellular carcinoma [24], breast cancer [25], esophageal squamous cell carcinoma [17], and bladder cancer [26]. Also, it is reported that CS could dysregulate *EYA4* expression [27]. Therefore, in the current study, we have investigated the effect of CS on DNA methylation level in nonsmoker and smoker Saudi adults as well as the contribution of DNA methylation in regulating *EYA4* expression.

## 2. Materials and Methods

### 2.1. Ethical Approval

The ethical approval of this study was obtained from the Research Ethics Committee of the College of Applied Medical Sciences at King Saud University in Riyadh, Saudi Arabia (Reference No. CAMS 13/3536).

### 2.2. Collection of Blood Samples

We have collected blood samples from 100 healthy Saudi adults of which 50 people are smokers and other 50 nonsmokers (Table 1), from the Blood Donation Center at King Saud medical city (Riyadh, Saudi Arabia) between September 2018 and December 2019.

### 2.3. DNA Extraction, Bisulfite Conversion, and Sanger Sequence

The lymphocyte genomic DNA was extracted with PureLink® Genomic DNA Mini Kit (Invitrogen) [28] and 500 ng was treated with EZ DNA methylation-Gold ™ kit (Zymo Research) [12]. *EYA4* forward AGGGGATGTTTTGTTTTTATTAGAG and reverse TAAAAATTCTCTCAACTCAAACTCC were amplified using end point PCR, PCR condition: 5 minutes at 95°C; followed by 37 cycles, 94°C for 30 seconds, and then 30 seconds at 60°C and 30 seconds at 72°C, respectively. Having terminated the amplification with a 10 minutes at 72°C, followed by sanger sequencing via Macrogen Inc. (Seoul, Republic of Korea).

### 2.4. Cells and 5-Aza-2′-Deoxycytidine Treatment

The LoVo and Caco-2 were obtained from American Type Culture Collection (ATCC), USA. Cells were grown in DMEM (Sigma) media containing 10% FBS and 10000 U/ml antibiotic and then kept at 37°C in 5% CO_2_ incubator. LoVo and Caco-2 were treated with 1 *μ*M 5-aza-2′-deoxycytidine (Sigma) for 72 hours, and a medium was replaced every 24 hours. Control cultures had an equal volumes of drug solvent (DMSO) [12].

### 2.5. RNA Extraction, cDNA Synthesis, and RT-PCR

Total RNA was extracted with a QIAZol Lysis reagent (Qiagen), and GoScript™ Reverse Transcritase (Promega) was applied to synthesis cDNA; gene-specific primers of *EYA4* forward ATAACACAGCCGATGGCACA and reverse TCCTGGTTGGTTAGTCAGTCC were used for QPCR (GoTaq® qPCR; Promega) on Prime Q real-time PCR machine (Techine), normalizing the amount of target gene to the house keeping gene *GAPDH* forward AATGGGCAGCCGTTAGGAAA and reverse AAAAGCATCACCCGGAGGAG [29]. PCR conditions are as follows: one cycle at 95°C for 15 minutes, followed by 36 cycles of 95°C for 30 seconds, then 30 seconds at 58°C and 30 seconds at 72°C, terminating the incubation by 1 cycle of 95°C for 1 minute, 58°C for 30 seconds, and 95°C for 30 seconds successively. The 2^−ΔΔCt^ method was applied to define the relative mRNA expression.

### 2.6. Statistical Analysis

Statistical analysis was performed using SPSS software Ver.22 (SPSS Inc., Chicago, USA). Data were examined using Student's *t*-test, and results were presented as average ± SD. Paired *t*-test were being considered statistically significant at ^∗^*p* < 0.05; ^∗∗^*p* < 0.005.

## 3. Results

### 3.1. Clinical Data of the Participants

In this study, there was no significant difference in the age of participants (average age nonsmokers = 29.85 years old and smokers = 31.75 years old) (Table 1). Smoker participants consume a minimum of 10 cigarettes a day for a minimum of 7 years.

### 3.2. *EYA4* Promoter Is Enriched with CpG Islands, and Its Expression Is Downregulated in Colon Cancer

We designed our assay on *EYA4* promoter region which is enriched with CpG island (on human genome build NCBI36/Hg18 (UCSC genome browser; http://genome.ucsc.edu) (Figure 1(a)). Also, we have noticed that the expression of *EYA4* is decreased in number of colon cancer sets: GSE8672, GSE4554, GSE2150, and GSE37892 compared to different set of normal tissues GSE3526 and GSE7307 that are appeared in R2 genomic analysis and visualization platform (https://hgserver1.amc.nl/cgi-bin/r2/main.cgi) (Figure 1(b)). These data suggested the possible relation between DNA methylation and regulation of *EYA4* expression.

### 3.3. *EYA4* Amplification in Bisulfite Genomic DNA Extracted from Smoker and Nonsmoker Adults

Genomic DNA was extracted from participants and was treated with bisulfite conversion, followed by PCR amplification. The expression of *EYA4* was detected in all samples (Figure 2). Then, PCR products were dispatched for Sanger sequence to see the alternation of DNA methylation level.

### 3.4. *EYA4* Methylation in Nonsmoker and Smoker Adults

Interestingly, Sanger sequence data has shown that there is no methylation on *EYA4* promoter in all nonsmoker samples (Figure 3(a)), However, 26% of smokers harbored methylated promoter of *EYA4* (Figure 3(b)). The level of DNA methylation was significantly increased in smokers compared to nonsmokers (Figure 3(c)). Our results indicated that CS causes a noticeable change in DNA methylation. Therefore, the effect of DNA methylation on the regulation of the *EYA4* expression was investigated in colon cancer cell lines.

### 3.5. 5-Aza-2′-Deoxycytidine Induces *EYA4* Expression

Colon cancer cell lines LoVo and Caco-2 were treated with 1 *μ*M 5-Aza-CdR for 72 hours, and the expression of *EYA4* was significantly upregulated in LoVo (Figure 4(a)) and Caco-2 (Figure 4(b)) compared to cells treated with DMSO.

Taken together, our results suggested that CS could epigenetically regulate the expression of *EYA4* through the alternation of DNA methylation.

## 4. Discussion

In this paper, we have examined the effect of CS on the regulation of DNA methylation as well as the involvement of DNA methylation in controlling the expression *EYA4* gene. The expression of *EYA4* gene is important in cell proliferation, migration, and angiogenesis [21]. *EYA4* promoter is covered with CpG island, and alternation of DNA methylation was observed in tumor samples compared to normal samples [17, 30]. Additionally, abnormality of *EYA4* expression has been mentioned to contribute to cancer progression for instance, colon cancer [31], glioma [32], lung cancer [23], and bladder cancer [26]. Also, downregulation of its expression was defined in different sets of colon cancers, suggesting its role in inhibiting tumor development [31]. A recent study by Deger et al. revealed the role of *EYA4* methylation in predicting the favourable outcomes of colorectal liver metastasis patients as the level of DNA methylation has comparably decreased in blood samples taken from patients after and before treatments [33].

Interestingly, our result showed for the first time among Saudi population, no methylation of *EYA4* was appeared in nonsmokers, whereas 26% of smoker samples were methylated and these differences are significant. Our finding is in line with that found in Zhu et al. [34] in DNA methylation of cigarette smoking of the Chinese population. Also, other researchers have reported that DNA methylation is associated with cigarette smoking [34–37], and changing the methylation in one CpG could induce gene expression [38]. Thus, due to the involvement of CS in alteration of DNA methylation status [39, 40], and in hampering the expression of *EYA4* in lung tissues taken from smokers compared to nonsmokers [27] as well as the impact of DNA methylation in depleting *EYA4* expression in oral [41] and colon cancer [31], we suggest that CS could have a role in changing the methylation status of *EYA4* in Saudi population.

CS is implicated in inducing hypermethylation mechanism via increasing the expression of DNA methyl transferase enzymes (DNMTs) [42, 43]. The possible mechanism could be through DNA damage on *DNMT3b* which occurs as a result of the existences of carcinogens content in CS including arsenic, formaldehyde, and nitrosamines [44], leading to a transition from C to T that is located on the promoter 149 bp away from the transcription start site; it was revealed that nonsmokers harbor *DNMT3b*–149 CT genotype while smokers contain *DNMT3b*–149 TT genotype [42]. Consequently, an increase of *DNMT3b* activity is observed, causing an establishment of de novo methylation of CpG on some tumor suppressor genes [45].

A few studies have shown the dysregulation of DNA methylation in colon cancer including *EYA4*, which was hypermethylated and treatment with demethylating agents caused induction of its expression [46]. In agreement with Kim et al. [31] and Moon et al. [47], we have restored the expression of *EYA4* after treating the Caco-2 and LoVo colon cancer cells with 1 *μ*M 5-Aza-CdR for 72 hours, this implies the possible mechanism of involvement of DNA methylation in hampering the expression of *EYA4* [31], which could accelerate colon cancer formation [31].

The consequence of the existence of *EYA4* expression conceivably blocks the development of colon cancer [31], through the downregulation of MYCBP [48] via dephosphorylating *β*-catenin [49]. Therefore, the depletion of *EYA4* expression has been detected in colorectal cancer, possibly due to hypermethylated promoter [31]. Overall, our result indicates the deleterious impacts of CS on the alternation of the level of DNA methylation in *EYA4* promoter, presumably resulting in *EYA4* inhibition.

## Figures and Tables

**Figure 1:** Location of *EYA4* assay and RNA expression in normal tissues and colon cancer. (a) USCS genome browser (https://genome.ucsc.edu) indicates the place of amplicon on the *EYA4* promoter and the distribution of CpG island on the promoter region of *EYA4*. (b) Box blot shows the expression of *EYA4* in normal tissues (1: GSE3526 contains 353 samples and 2: GSE7307 contains 504 samples) and in colon cancers (1: GSE8671 contains 32 samples, 2: GSE4554 contains 84 samples, 3: GSE21510 contains 148 samples, and 4: GSE37892 contains 130 samples) taken from R2 online public data (https://hgserver1.amc.nl/cgi-bin/r2/main.cgi).

**Figure 2:** 2% agarose gel of PCR product shows the amplification of *EYA4* gene in lymphocyte genomic DNA extracted from nonsmokers and smokers. Followed by treatment with bisulfite conversion in nonsmoker and smoker adults. 1 to 50 indicates the samples number. (a) *EYA4* bands after being amplified by PCR in 50 samples of nonsmokers. (b) *EYA4* bands after being amplified by PCR in 50 samples of smokers.

**Figure 3:** *EYA4* methylation level in nonsmoker and smoker samples. (a) Lollipop diagram displays the methylation level of 4 CpG islands that located on the EYA4 promoter in DNA extracted from nonsmokers (*n* = 50). White lollipop indicates unmethylated cytosine, black lollipop indicates methylated cytosine, and there was no methylation observed. (b) Lollipop diagram displays the methylation level of 4 CpG islands that located on the EYA4 promoter in DNA extracted from nonsmokers (*n* = 50). White lollipop indicates unmethylated cytosine, black lollipop indicates methylated cytosine, and methylated cytosine was detected in 26% of tested samples. (c) Box blot shows the number of methylated cytosine in nonsmoker and smoker adults. ^∗∗^*p* < 0.01, two samples *t*-test.

**Figure 4:** The effects of 5-Aza-CdR on *EYA4* RNA expression in colon cancer cells. (a) RNA expression of *EYA4* in Caco-2 cell lines after being treated with DMSO (control) and with 1 *μ*M 5-Aza-CdR (AZA) for 72 hours and media was replaced every 24 hours. (b) RNA expression of *EYA4* in LoVo cell lines after being treated with DMSO (control) and with 1 *μ*M 5-Aza-CdR (AZA) for 72 hours and media was replaced every 24 h. Mean ± SD of three experiments, ^∗^*p* < 0.05, ^∗∗^*p* < 0.005, paired sample *t*-test.

**Table 1:** Clinical and demographic data of the study participants.

Variable	Smokers	Nonsmokers
Number	50	50
Age (years), median ± SD	31.75 ± 2.84	29.8 ± 3.5
Age (years)		
≤30 years	31 (62%)	18 (36%)
>30 years	19 (38%)	32 (64%)
Years of smoking		
≤12 years	26 (52%)	—
>12 years	24 (48%)	—

## Data Availability

The original contributions presented in the study are included in the article; further inquiries can be directed to the corresponding author.
